# Increased Serum Levels of sCD206 Are Associated with Adverse Prognosis in Patients with HBV-Related Decompensated Cirrhosis

**DOI:** 10.1155/2022/7881478

**Published:** 2022-05-25

**Authors:** Yue Zhang, Nanxi Xiao, Qi Liu, Yuan Nie, Xuan Zhu

**Affiliations:** Department of Gastroenterology, Jiangxi Clinical Research Center for Gastroenterology, The First Affiliated Hospital of Nanchang University, Nanchang, Jiangxi, China

## Abstract

**Background:**

HBV-associated decompensated cirrhosis (HBV-DeCi) is attracting considerable attention due to disease acceleration and substantial mortality. Macrophages regulate the fibrotic process in DeCi. Soluble CD206 (sCD206) is primarily expressed by macrophages. We aimed to investigate whether sCD206 predicts mortality in patients with HBV-DeCi.

**Materials and Methods:**

A total of 382 patients were enrolled between February 2020 and February 2021 and divided into nonsurviving and surviving groups according to 28-day, 3-month, and 6-month outcomes. Cox regression analysis was performed to confirm the independent prognostic factors of HBV-DeCi, and Kaplan–Meier analysis was performed to draw survival curves of sCD206. The predictive value of sCD206 was assessed at three time points according to the AUROC.

**Results:**

The serum sCD206 level was significantly higher in deceased patients than surviving patients. Multivariate analysis showed that the level of sCD206 was related to an increased risk of 28-day, 3-month, and 6-month mortality (HR = 3.914, *P* < 0.001; HR = 3.895, *P* < 0.001; and HR = 4.063, *P* < 0.001, respectively). Patients with higher sCD206 levels had a worse prognosis than those with lower sCD206 levels. The best separation between the decedents and survivors was obtained by using the sCD206 level (AUROC: 0.830, 0.802, and 0.784, respectively) at 28 days, 3 months, and 6 months.

**Conclusion:**

The macrophage-related marker serum sCD206 was associated with mortality in HBV-DeCi patients. High levels of serum sCD206 indicated a poor prognosis in these patients. Serum sCD206 has great predictive value for short-term and midterm mortality compared with the Child-Turcotte-Pugh (CTP) and model for end-stage liver disease (MELD) scores.

## 1. Introduction

Hepatitis B virus (HBV) infection is a serious global health problem; approximately 257 million people worldwide are chronic HBV surface antigen (HBsAg) carriers, of whom 78 million reside in China [1]. HBV infection is related to acute and chronic liver hepatitis, liver cirrhosis, and hepatocellular carcinoma (HCC) [2]. Decompensated cirrhosis (DeCi) is a common and serious liver disease that develops mainly in chronic hepatitis B (CHB) patients in Asia and is a disease state in which patients with cirrhosis develop variceal bleeding, ascites, hepatic encephalopathy (HE), or jaundice [3]. Once decompensation occurs, cirrhosis becomes a systemic disease with multiorgan dysfunction [4]. The median survival time drops from more than 12 years for the compensated state to approximately 2 years for the decompensated state due to these events [5]. The only curative therapy for DeCi is liver transplantation [6]. However, the shortage of inadequate social support and donor livers has limited the clinical application of liver transplantation. Therefore, it is crucial to screen patients with a high mortality risk as early as possible, which can help tailor the treatment strategy, early intervention, or even early transfer to an intensive care unit.

Activated macrophages are associated with the pathogenesis of liver fibrosis [7]. Macrophages can be activated under the stimulation of chronic and acute inflammatory reactions, and they are polarized into M1 and M2 macrophages [8]. CD206, a mannose receptor, is primarily expressed on the surface of macrophage cells, where it acts as a pattern recognition receptor [9]. Soluble CD206 (sCD206) is the soluble form of CD206, and the plasma concentration of sCD206 is increased in liver cirrhosis [10, 11]. An increase in the soluble levels of CD206 has been confirmed to be a circulating marker of monocyte/macrophage activation in cirrhosis patients [11], and the shedding of sCD206 is promoted by pathogen-associated molecular patterns (PAMPs), including lipopolysaccharide [12]. In this study, we tested serological levels of sCD206 in HBV-DeCi patients and assessed whether serum sCD206 had an association with the mortality of such patients.

## 2. Materials and Methods

### 2.1. Study Population

We assessed 382 patients diagnosed with HBV-DeCi at the First Affiliated Hospital of Nanchang University between February 2020 and February 2021. All patients were hospitalized for acute decompensation events. The research was approved by the Ethics Committee of our institution and was consistent with the Declaration of Helsinki. Written informed consent was obtained from all patients. The inclusion criteria were as follows: patients (1) were more than 18 years old, (2) were hepatitis B surface antigen positive for longer than 6 months, (3) were diagnosed with decompensated cirrhosis, and (4) had available follow-up data. The exclusion criteria were as follows: (1) patients with alcoholic liver disease, drug-induced liver injury, autoimmune hepatitis, or other viral infections (hepatitis A, C, or E or HIV infections); (2) complications with hepatocellular carcinoma; (3) complications with other malignancies; and (4) no specific test results.

### 2.2. Definitions

The diagnosis of CHB was based on HBsAg positivity or detectable HBV DNA for more than six months. The diagnosis of DeCi was defined by radiologic evidence, biochemical results, or biopsy, including complications of cirrhosis, such as ascites, gastrointestinal bleeding, HE, spontaneous bacterial peritonitis (SBP), or hepatorenal syndrome. The Child-Turcotte-Pugh (CTP) score was calculated based on prothrombin time (PT), ascites, levels of albumin and serum bilirubin, and HE [13]. The model for end-stage liver disease (MELD) score was computed based on the formula: MELD = 9.6 × ln [serum creatinine (Scr) (mg/dl)] + 3.8 × ln [total bilirubin (mg/dl)] + 11.2 × ln [prothrombin time (international normalized ratio (INR))] + 6.43 × (etiology : 0 if cholestatic or alcoholic, 1 otherwise) [14]. The diagnosis and grading of ascites were defined according to the criteria proposed by the International Ascites Club [15]. HE was classified according to the practice guidelines of the European Association for the Study of the Liver (EASL) and American Association for the Study of Liver (AASLD) [16].

### 2.3. Determination of Plasma sCD206 Levels

Serum samples were stored at −80°C after collection from centrifuged peripheral blood. The sCD206 levels were determined using an enzyme-linked immunosorbent assay (ELISA) kit (RayBiotech, Norcross, GA, USA) according to the manufacturer's instructions.

### 2.4. Study Protocols

Physical examination, laboratory test, demographic, treatment history, and radiological examination data were acquired from electronic medical records. All blood tests were measured within 24 hours of admission. The sCD206 results were collected from a datasheet generated by laboratory professional staff. Overall survival (OS) was defined as the duration from admission to death or the last follow-up time (6 months).

### 2.5. Management of Patients

DeCi resulting from HBV was immediately treated with nucleoside analogs (entecavir alone 0.5 mg, lamivudine alone 100 mg, telbivudine alone 600 mg, or lamivudine 100 mg plus adefovir 10 mg daily). Patients with acute variceal bleeding were managed according to the Baveno VI consensus guidelines [17]. Patients with bacterial infection were immediately treated with empirical antibiotic therapy, and the adjustment of antibiotic therapy was based on bacterial culture and antibiotic sensitivity tests.

### 2.6. Statistical Analysis

Statistical analysis was conducted with the SPSS version 24.0 for Windows (SPSS, Inc., Chicago, IL) and the R software version 4.0.3 (The R Foundation for Statistical Computing, http://www.R-project.org), and ROC analysis was performed by using the MedCalc statistical software version 15.2.1 (MedCalc, Ostend, Belgium). Continuous variables with normal distributions were analyzed by the mean (SD) and compared using Student's *t*-test. Continuous variables without normal distributions were analyzed by medians (quartiles) and compared using the Mann–Whitney test. Categorical variables were compared using the chi-squared test or Fisher's exact test. A multivariable Cox regression model was applied to identify predictive factors for overall survival, including both correlated predictive factors at univariable analysis (*P* < 0.050) and clinically relevant variables. The survival curves were calculated using the “rms,” “survminer,” and “survival” packages in the R software, of which the ggsurvplot function was used to perform the K-M survival curve. The ROC curves were calculated using the “survminer,” “survival,” “timeROC,” and “pROC” packages in the R software. The Delong test was used to compare the AUROCs by the MedCalc software. The reported statistical significance levels were all two-sided, with significance set at 0.050.

## 3. Results

### 3.1. Demographic and Clinical Features

As depicted in Figure 1, according to the criteria set at the beginning of our study, we finally included 382 patients who were diagnosed with HBV-DeCi. The demographic and clinical features of the included patients are shown in Table 1. Among the 382 patients, 293 (76.7%) were males, and 89 (23.3%) were females. The main cause of decompensation events related hospitalization was gastrointestinal bleeding (247/382, 64.66%), ascites (57/382, 14.92%), infection (51/382, 13.35%), and hepatic encephalopathy (27/382, 7.07%). A total of 32 patients developed HE during their hospitalization, and the HE grade was 2nd degree HE (3.7%), followed by 3rd degree HE (2.3%), 4th degree HE (1.6%), and 1st degree HE (0.8%). The grade of ascites during hospitalization was mild (28.8%), moderate (14.4%), or severe (13.1%). Across the entire study population, 33.2% of the patients received vasopressor support. The sCD206 levels ranged from 0.26 to 0.58 mg/L (median: 0.36 mg/L). Among these patients, 48 patients died within 28 days, 77 patients died within 3 months, and 95 patients died within 6 months.

### 3.2. Clinical Characteristics of the Nonsurviving and Surviving Groups

The clinical characteristics of the nonsurviving and surviving patients with HBV-DeCi are shown in Table 2. HBV-DeCi patients were distributed into nonsurviving and surviving groups according to their 28-day, 3-month, and 6-month outcomes. The two groups significantly differed in bilirubin level, WBC count, PT, INR, levels of creatinine, ALT, AST, albumin, GGT, and ALP, CTP score, MELD score, and sCD206 level at all time points (all *P* < 0.050). Compared to the surviving group, the nonsurviving group had a higher bilirubin level, WBC count, PT, INR, level of creatinine, ALT, AST, GGT, and ALP, CTP score, MELD score, and sCD206 level and a lower albumin level (all *P* < 0.050). No significant differences in platelet counts or levels of MAP, PO_2_/FiO_2_, or serum sodium were observed at any follow-up time (*P* > 0.050).

### 3.3. Prognostic Factors in HBV-DeCi Patients

In univariable regression analysis, ten variables, i.e., age, the usage of vasopressors, creatinine, bilirubin, INR, WBC, PT, ALP, albumin, and sCD206, were significantly associated with overall survival at all follow-up times. All the significant factors found in the univariate analysis were included in the multivariable Cox regression analysis; the result revealed that the four variables, i.e., creatinine, ALP, albumin, and sCD206, were identified as independent prognostic factors of HBV-DeCi at any time point (Table 3, Figure 2).

### 3.4. The Prognostic Value of sCD206 Expression in HBV-DeCi Patients

As shown in Figure 3, Kaplan–Meier analysis was performed to evaluate sCD206 in HBV-DeCi patients, and patients with high sCD206 expression had a poorer prognosis than those with low sCD206 expression (*P* < 0.001). The cutoff value of sCD206 was 0.621 according to the data analysis.

### 3.5. sCD206 as a Prognostic Marker in HBV-DeCi Patients

The predictive ability of sCD206 was analyzed by receiver operating characteristic (ROC) curve analysis. The area under the ROC curve (AUCROC) of sCD206 was 0.830 (95% CI: 0.789–0.866), 0.802 (95% CI: 0.758–0.841), and 0.784 (95% CI: 0.739–0.824) for predicting survival probability at 28 days, 3 months, and 6 months, respectively (Table 4, Figure 4). As shown in Table 5, the predictive performance of sCD206 was significantly higher than that of the CTP and MELD scores at all time points (*P* < 0.050). The comparisons of the AUROC between sCD206 and the two scores are shown in Figure 5.

## 4. Discussion

Our study demonstrated that the serum sCD206 level was increased significantly in HBV-DeCi patients and that it helped distinguish nonsurvivors from survivors. sCD206 was an independent risk factor for the prognosis of such patients, and it has better performance than the CTP and MELD scores for predicting outcomes in HBV-DeCi patients.

As described previously, DeCi is marked by the development of overt clinical signs, the most frequent of which are bleeding, ascites, jaundice, and encephalopathy. Once these signs occur, the disease usually progresses more rapidly toward liver transplantation (LT) and even death. Therefore, the grave prognosis in HBV-DeCi patients mandates the identification of better prognostic indicators. At present, many prognostic models have been used to predict the outcome of DeCi patients, such as the CTP score and MELD score. The CTP score is easy to calculate but includes two subjective variables, namely, HE and ascites. A previous study showed that the MELD score had good accuracy in predicting mortality in DeCi patients [18]; however, these scores do not contain markers that reflect disease progression or pathogenesis, so identifying new markers that can effectively predict outcome is necessary.

Liver macrophages represent >80% of the total macrophage population and play a key role in the development and progression of liver inflammation and fibrosis [19, 20]. Macrophage activation by pathogen-associated molecular patterns (PAMPs) and damage-associated molecular patterns (DAMPs), interferon-*γ* (IFN-*γ*), and the cytokine interleukin-12 (IL-12) are known to produce a proinflammatory response in macrophages, resulting in the release of IL-1*β*, IL-6, IL-12, tumor necrosis factor (TNF), and reactive oxygen species [21, 22]. Moreover, the presence of an IFNL3-IFNL4 haplotype resulting in the production of IFN-*γ*3 is considered a promoter of fibrosis progression and hepatic inflammation [23]. CD163 was the hemoglobin-haptoglobin scavenger receptor highly expressed by macrophages; our previous study had confirmed that the plasma soluble CD163 had well predictive value in predicting outcome in DeCi patients [24]. As the other scavenger receptor, CD206 is also highly expressed by macrophages and is known as the mannose receptor [25]. CD206 is the soluble form and exists in culture media from human dendritic cells, human macrophages, and human serum [26]. As a macrophage activation marker, sCD206 mediates a series of immune responses that recognize, phagocytose, and clear pathogens. A recent study showed that the levels of serum sCD206 stemmed from liver macrophages [26]. sCD206 may play important roles in the immune process of serious disease. Zou et al. found that the macrophage activation marker sCD206 was associated with the mortality of idiopathic pulmonary fibrosis patients [27]. Recently, it was confirmed that sCD206 was elevated in patients with acute-on-chronic liver failure (ACLF) and related to disease severity [28]. Previous studies have shown that sCD206 is significantly elevated in patients with cirrhosis compared to healthy individuals and increases with increased liver disease severity, and among patients with alcoholic cirrhosis, the sCD206 level predicts portal hypertension [12]. If portal pressure exceeds a certain threshold, the patient is at risk of developing life-threatening bleeding from varices. In addition, a previous study showed that CD206 expresses amphiregulin to promote regulatory T-cell activity and subsequently restrain CD8 T-cell-mediated antiviral function in a mouse HBV model, which may accelerate disease progression [29]. Importantly, sCD206 is stable during freezing and thawing and easily obtainable, and both commercial and house ELISAs are available, which makes them ideal biomarkers for use in daily clinical practice.

Our study has several limitations. First, a validated cohort was lacking to confirm the findings. Second, the dynamic changes in serum sCD206 should be determined during the progression of HBV-DeCi. Third, multicenter studies with large sample sizes are required to confirm the current findings.

In conclusion, serum sCD206 levels are significantly elevated in nonsurviving HBV-DeCi patients, and sCD206 expression may be a crucial prognostic indicator in such patients. In addition, sCD206 has better discriminative power than MELD or Child-Pugh score for assessing short-term and midterm mortality. The present findings collectively suggest that the sCD206 level may be a predictor of prognosis in patients with HBV-DeCi.

## Figures and Tables

**Figure 1:** Flowchart of the selection of patients with HBV-DeCi.

**Figure 2:** The constitution of the multivariable Cox model is shown as a forest plot: (a) 28 days; (b) 3 months; (c) 6 months.

**Figure 3:** Kaplan–Meier survival analysis shows the relationship of sCD206 expression.

**Figure 4:** ROC curve analysis of sCD206 for predicting 28-day, 3-month, and 6-month mortality.

**Figure 5:** ROC curve analysis between sCD206 and two scores for predicting 28-day, 3-month, and 6-month mortality: (a) ROC for 28 days; (b) ROC for 3 months; (c) ROC for 6 months.

**Table 1:** Baseline clinical and laboratory characteristics of patients with HBV-DeCi.

	HBV-DeCi patients (*n* = 382)
Sex, *n* (%)	
Male	293 (76.70)
Female	89 (23.30)
Age, mean ± SD, years	54.55 ± 11.78
Cause of admission, *n* (%)	
Gastrointestinal bleeding	247 (64.66)
Ascites	57 (14.92)
Infection	51 (13.35)
Hepatic encephalopathy	27 (7.07)
Hepatic encephalopathy degree, *n* (%)	
1st degree HE	3 (0.80)
2nd degree HE	14 (3.70)
3rd degree HE	9 (2.30)
4th degree HE	6 (1.60)
Ascites degree, *n* (%)	
Mild	110 (28.80)
Moderate	55 (14.40)
Severe	50 (13.10)
Vasopressor support, *n* (%)	127 (33.20)
Biochemical parameters	
WBC, 10^∗^9/L	6 (4-10)
Platelet, 10^∗^9/L	64 (41-95)
PT, s	14.90 (13.60-16.8)
INR	1.33 (1.21-1.53)
Bilirubin, *u*mol/L	24.00 (15.75-39.00)
ALT, IU/L	26.00 (18.00-45.00)
AST, IU/L	41.00 (28.00-76.00)
sCD206	0.36 (0.26-0.58)
CTP score	8.00 (7.00-10.00)
MELD score	11.00 (9.00-14.00)

HBV: hepatitis B virus; SD: standard deviation; HE: hepatic encephalopathy; WBC: white blood cell count; PT: prothrombin time; INR: international normalized ratio; ALT: alanine aminotransferase; AST: aspartate aminotransferase; sCD206: soluble CD206; CTP: Child-Turcotte-Pugh; MELD: model for end-stage liver disease.

**Table 2:** The comparison of clinical characteristics between nonsurviving and surviving patients.

Variables	28 days		*P* value	3 months		*P* value	6 months		*P* value
	Nonsurvivors (*n* = 48)	Survivors (*n* = 334)		Nonsurvivors (*n* = 77)	Survivors (*n* = 305)		Nonsurvivors (*n* = 95)	Survivors (*n* = 287)	
Bilirubin, *μ*mol/L	26.00 (15.25-73.25)	23.00 (15.75-37.00)	*<0.001*	26.00 (17.00-54.50)	23.00 (15.00-36.00)	*<0.001*	27.00 (18.00-59.00)	22.00 (15.00-36.00)	*<0.001*
Platelet, 10^∗^9/L	62.00 (41.00-93.00)	72.00 (36.00-117.00)	0.168	62.00 (41.50-92.00)	76.00 (37.50-116.50)	0.123	62.00 (41.00-92.00)	70.50 (42.75-115.00)	0.087
WBC, 10^∗^9/L	9.00 (5.00-15.00)	6.00 (4.00-9.00)	*0.001*	8.00 (5.00-14.00)	6.00 (4.00-9.00)	*0.001*	8.00 (5.00-12.00)	6.00 (4.00-9.00)	*0.003*
PT	15.10 (13.90-21.05)	14.80 (13.55-16.50)	*0.016*	15.50 (13.95-20.80)	14.80 (13.43-16.40)	*0.001*	15.40 (13.90-19.90)	14.80 (13.38-16.40)	*0.002*
INR	1.44 (1.24-1.81)	1.32 (1.20-1.49)	*0.001*	1.44 (1.26-1.82)	1.31 (1.19-1.48)	*<0.001*	1.39 (1.24-1.75)	1.31 (1.19-1.48)	*0.001*
Creatinine, *μ*mol/L	103.00 (70.50-142.25)	71.00 (58.00-86.00)	*<0.001*	89.00 (62.50-136.00)	71.00 (58.00-85.00)	*<0.001*	86.00 (62.00-134.00)	70.00 (57.00-84.00)	*<0.001*
ALT, IU/L	37.50 (17.25-87.25)	26.00 (18.00-41.25)	*0.012*	37.00 (18.50-91.50)	25.00 (18.00-40.50)	*0.006*	37.00 (18.00-84.00)	25.00 (18.00-39.00)	*0.005*
AST, IU/L	80.50 (39.50-198.25)	39.00 (27.00-67.25)	*<0.001*	79.00 (39.00-214.00)	37.00 (27.00-59.50)	*<0.001*	68.00 (37.00-190.00)	37.00 (26.00-58.00)	*<0.001*
MAP, mmHg	81.50 (76.25-87.75)	83.00 (78.00-88.00)	0.307	83.00 (78.00-88.00)	83.00 (78.00-88.20)	0.876	83.00 (79.00-88.00)	83.00 (78.00-88.00)	0.638
PO2/FiO2	395.13 ± 115.03	419.65 ± 116.64	0.116	394.75 ± 122.60	418.93 ± 115.52	0.106	398.04 ± 122.87	419.36 ± 115.02	0.125
Albumin, g/L	25.33 ± 4.70	28.70 ± 7.89	*<0.001*	25.35 ± 5.15	29.02 ± 7.99	*<0.001*	25.69 ± 4.97	29.13 ± 8.17	*<0.001*
Serum sodium	137.00 (134.00-143.75)	138.00 (136.00-141.00)	0.956	138.00 (134.00-142.00)	138.00 (136.00-141.00)	0.585	138.0 (135.00-141.00)	138.00 (136.00-141.00)	0.644
GGT, IU/L	45.50 (18.00-92.75)	22.00 (13.00-46.00)	*0.001*	39.00 (18.00-95.50)	22.00 (13.00-46.00)	*0.001*	37.00 (16.00-83.00)	22.00 (13.00-46.00)	*0.004*
ALP, IU/L	93.00 (59.25-159.75)	67.00 (52.00-96.25)	*0.002*	83.00 (52.00-162.00)	67.00 (53.00-93.50)	*0.004*	82.00 (56.00-154.00)	67.00 (52.00-93.00)	*0.002*
CTP score	10.00 (8.00-10.75)	8.00 (7.00-9.00)	*<0.001*	9.00 (8.00-10.00)	8.00 (7.00-9.00)	*<0.001*	9.00 (8.00-10.00)	8.00 (7.00-9.00)	*<0.001*
MELD score	15.00 (10.00-22.75)	11.00 (9.00-14.00)	*<0.001*	15.00 (11.00-20.00)	11.00 (9.00-13.00)	*<0.001*	14.00 (10.00-19.00)	10.00 (9.00-13.00)	*<0.001*
sCD206, mg/L	0.86 (0.49-1.78)	0.34 (0.24-0.49)	*<0.001*	0.65 (0.42-1.17)	0.24 (0.19-0.34)	*<0.001*	0.64 (0.38-1.05)	0.34 (0.24-0.43)	*<0.001*

*P* value < 0.05 was considered significant and was indicated in italic. WBC: white blood cell count; PT: prothrombin time; INR: international normalized ratio; ALT: alanine aminotransferase; AST: aspartate aminotransferase; MAP: mean arterial pressure; GGT: gamma-glutamyl transpeptidase; ALP: alkaline phosphatase; CTP: Child-Turcotte-Pugh; MELD: model for end-stage liver disease; sCD206: soluble CD206.

**Table 3:** Univariate and multivariate analyses of clinical variables at 28-day, 3-month, and 6-month follow-ups.

	28 days				3 months				6 months			
	Univariate		Multivariate		Univariate		Multivariate		Univariate		Multivariate	
	HR (95% CI)	*P* value	HR (95% CI)	*P* value	HR (95% CI)	*P* value	HR (95% CI)	*P* value	HR (95% CI)	*P* value	HR (95% CI)	*P* value
Sex												
Female	Reference				Reference				Reference			
Male	1.229 (0.650-2.322)	0.526			1.014 (0.598-1.719)	0.959			0.882 (0.538-1.444)	0.617		
Age												
<60	Reference				Reference				Reference			
≥60	2.142 (1.216-3.771)	*0.008*			1.851 (1.182-2.900)	*0.007*			1.711 (1.140-2.568)	*0.010*		
The usage of vasopressor												
No using	Reference				Reference				Reference			
Using	2.726 (1.541-4.821)	*0.001*			1.932 (1.235-3.024)	*0.004*			1.687 (1.124-2.533)	*0.012*		
Platelet, 10^∗^9/L	1.003 (0.999-1.005)	0.116			1.003 (1.000-1.005)	0.151			1.003 (1.000-1.007)	0.058		
Creatinine, *μ*mol/L	1.009 (1.007-1.012)	*<0.001*	1.009 (1.004-1.013)	*<0.001*	1.009 (1.007-1.011)	*<0.001*	1.008 (1.005-1.012)	*<0.001*	1.009 (1.007-1.012)	*<0.001*	1.008 (1.005-1.012)	*<0.001*
Bilirubin, *μ*mol/L	1.010 (1.007-1.013)	*<0.001*			1.009 (1.006-1.012)	*<0.001*			1.009 (1.006-1.011)	*<0.001*		
INR	2.338 (1.598-3.422)	*<0.001*			2.402 (1.752-3.294)	*<0.001*			2.258 (1.653-3.086)	*<0.001*		
WBC, 10^∗^9/L	1.046 (1.021-1.072)	*<0.001*			1.039 (1.016-1.062)	*0.001*			1.032 (1.010-1.055)	*<0.001*		
PT	1.075 (1.030-1.122)	*0.001*			1.078 (1.042-1.115)	*<0.001*			1.071 (1.037-1.106)	*<0.001*		
PO_2_/FiO_2_	0.997 (0.994-1.001)	0.061			0.998 (0.996-1.000)	0.072			0.998 (0.997-1.000)	0.083		
MAP, mmHg	0.983 (0.955-1.012)	0.240			1.000 (0.977-1.024)	0.999			1.004 (0.983-1.026)	0.690		
AST, IU/L	1.000 (1.000-1.001)	0.112			1.000 (1.000-1.001)	0.097			1.000 (1.000-1.001)	0.106		
ALT, IU/L	1.000 (1.000-1.001)	0.169			1.000 (1.000-1.001)	0.242			1.000 (1.000-1.001)	0.185		
ALP, IU/L	1.004 (1.002-1.007)	*0.001*	1.004 (1.001-1.007)	*0.008*	1.004 (1.002-1.006)	*<0.001*	1.004 (1.002-1.007)	*0.001*	1.003 (1.001-1.005)	*0.001*	1.004 (1.001-1.006)	*0.002*
GGT, IU/L	1.002 (0.999-1.003)	0.072			1.001 (1.000-1.003)	0.063			1.001 (1.000-1.003)	0.153		
Serum sodium, mmol/L	1.021(0.969-1.076)	0.435			1.012 (0.978-1.047)	0.4813			1.013 (0.982-1.044)	0.425		
Albumin, g/L	0.881 (0.830-0.935)	*<0.001*	0.977 (0.916-0.987)	*0.045*	0.875 (0.834-0.918)	*<0.001*	0.950 (0.902-0.999)	*0.049*	0.885 (0.847-0.924)	*<0.001*	0.950 (0.906-0.995)	*0.030*
sCD206, mg/L	4.147 (3.103-6.332)	*<0.001*	3.914 (2.419-4.472)	*<0.001*	4.177 (3.206-5.443)	*<0.001*	3.895 (2.576-5.889)	*<0.001*	4.147 (3.209-5.359)	*<0.001*	4.063 (2.755-5.990)	*<0.001*

*P* value < 0.05 was considered significant and was indicated in italic. INR: international normalized ratio; WBC: white blood cell count; PT: prothrombin time; MAP: mean arterial pressure; AST: aspartate aminotransferase; ALT: alanine aminotransferase; ALP: alkaline phosphatase; GGT: gamma-glutamyl transpeptidase; sCD206: soluble CD206.

**Table 4:** The efficacy of sCD206 and prognostic scores for predicting mortality in 28 days, 3 months, and 6 months.

Prognostic score	AUROC	95% CI	*P* value	Cut-off point	Sensitivity (%)	Specificity (%)	PPV (%)	NPV (%)
28-day mortality								
CTP score	0.702	0.654-0.748	*<0.0001*	9	56.25	79.04	27.83	92.63
MELD score	0.672	0.623-0.719	*0.0007*	19	35.42	96.11	56.68	91.19
sCD206	0.830	0.789-0.866	*<0.0001*	0.413	85.42	68.26	27.89	97.02
3-month mortality								
CTP score	0.679	0.630-0.726	*<0.0001*	8	62.34	64.59	30.77	87.17
MELD score	0.711	0.663-0.756	*<0.0001*	13	59.74	76.07	38.66	88.21
sCD206	0.802	0.758-0.841	*<0.0001*	0.470	71.43	77.70	44.71	91.51
6-month mortality								
CTP score	0.685	0.635-0.731	*<0.0001*	8	62.11	66.20	37.82	84.07
MELD score	0.702	0.654-0.748	*<0.0001*	14	49.47	83.62	49.99	83.33
sCD206	0.784	0.739-0.824	*<0.0001*	0.621	71.58	72.47	46.26	88.51

*P* value < 0.05 was considered significant and was indicated in italic. AUROC: area under the receiver operating characteristic; PPV: positive predictive values; NPV: negative predictive values; CTP: Child-Turcotte-Pugh; MELD: model for end-stage liver disease. sCD206: soluble CD206.

**Table 5:** The comparison of predictive value between sCD206 and scores.

Prognostic score	Difference between areas (95% CI)	*P* value
28-day mortality		
sCD206 vs. CTP	0.1280 (0.0362-0.2200)	*0.006*
sCD206 vs. MELD	0.1580 (0.0454-0.2700)	*0.006*
3-month mortality		
sCD206 vs. CTP	0.1230 (0.0449-0.2000)	*0.002*
sCD206 vs. MELD	0.0905 (0.00177-0.1790)	*0.040*
6-month mortality		
sCD206 vs. CTP	0.0994 (0.0269-0.1720)	*0.007*
sCD206 vs. MELD	0.0816 (0.00114-0.1620)	*0.047*

*P* value < 0.05 was considered significant and was indicated in italic. CTP: Child-Turcotte-Pugh; MELD: model for end-stage liver disease; sCD206: soluble CD206.

## Data Availability

The data that support the findings of this study are available from the corresponding author, X.Z., upon reasonable request.

## References

[1] Zhang S., Wang F., Zhang Z. (2017). Current advances in the elimination of hepatitis B in China by 2030. *Frontiers of Medicine*.

[2] Iannacone M., Guidotti L. G. (2022). Immunobiology and pathogenesis of hepatitis B virus infection. *Nature Reviews Immunology*.

[3] Gines P., Krag A., Abraldes J. G., Sola E., Fabrellas N., Kamath P. S. (2021). Liver cirrhosis. *Lancet*.

[4] D'Amico G., Bernardi M., Angeli P. (2022). Towards a new definition of decompensated cirrhosis. *Journal of Hepatology*.

[5] D'Amico G., Garcia-Tsao G., Pagliaro L. (2006). Natural history and prognostic indicators of survival in cirrhosis: a systematic review of 118 studies. *Journal of Hepatology*.

[6] Shiffman M. L. (2020). Approach to the patient with chronic hepatitis B and decompensated cirrhosis. *Liver International: Official Journal of the International Association for the Study of the Liver*.

[7] Cardoso C. C., Matiollo C., Pereira C. H. J. (2021). Patterns of dendritic cell and monocyte subsets are associated with disease severity and mortality in liver cirrhosis patients. *Scientific Reports*.

[8] Shapouri-Moghaddam A., Mohammadian S., Vazini H. (2018). Macrophage plasticity, polarization, and function in health and disease. *Journal of Cellular Physiology*.

[9] Gantzel R. H., Kjaer M. B., Laursen T. L. (2021). Macrophage activation markers, soluble CD163 and mannose receptor, in liver fibrosis. *Frontiers in Medicine*.

[10] Laursen T. L., Wong G. L., Kazankov K. (2018). Soluble CD163 and mannose receptor associate with chronic hepatitis B activity and fibrosis and decline with treatment. *Journal of Gastroenterology and Hepatology*.

[11] Nielsen M. C., Andersen M. N., Rittig N. (2019). The macrophage-related biomarkers sCD163 and sCD206 are released by different shedding mechanisms. *Journal of Leukocyte Biology*.

[12] Sandahl T. D., Stoy S. H., Laursen T. L. (2017). The soluble mannose receptor (sMR) is elevated in alcoholic liver disease and associated with disease severity, portal hypertension, and mortality in cirrhosis patients. *PLoS One*.

[13] Pugh R. N., Murray-Lyon I. M., Dawson J. L., Pietroni M. C., Williams R. (2005). Transection of the oesophagus for bleeding oesophageal varices. *The British Journal of Surgery*.

[14] Kamath P. S., Wiesner R. H., Malinchoc M. (2001). A model to predict survival in patients with end-stage liver disease. *Hepatology*.

[15] Moore K. P., Wong F., Gines P. (2003). The management of ascites in cirrhosis: report on the consensus conference of the International Ascites Club. *Hepatology*.

[16] (2014). Hepatic encephalopathy in chronic liver disease: 2014 practice guideline by the European Association for the Study of the Liver and the American Association for the Study of Liver Diseases. *Journal of Hepatology*.

[17] de Franchis R., Baveno V. I. F. (2015). Expanding consensus in portal hypertension: report of the Baveno VI Consensus Workshop: stratifying risk and individualizing care for portal hypertension. *Journal of Hepatology*.

[18] Jepsen P., Watson H., Macdonald S., Vilstrup H., Jalan R. (2020). MELD remains the best predictor of mortality in outpatients with cirrhosis and severe ascites. *Alimentary Pharmacology & Therapeutics*.

[19] Boltjes A., Movita D., Boonstra A., Woltman A. M. (2014). The role of Kupffer cells in hepatitis B and hepatitis C virus infections. *Journal of Hepatology*.

[20] Ishibashi H., Nakamura M., Komori A., Migita K., Shimoda S. (2009). Liver architecture, cell function, and disease. *Seminars in Immunopathology*.

[21] Medzhitov R. (2008). Origin and physiological roles of inflammation. *Nature*.

[22] Tacke F., Zimmermann H. W. (2014). Macrophage heterogeneity in liver injury and fibrosis. *Journal of Hepatology*.

[23] Eslam M., McLeod D., Kelaeng K. S. (2017). IFN-lambda 3, not IFN-lambda 4, likely mediates IFNL3-IFNL4 haplotype-dependent hepatic inflammation and fibrosis. *Nature Genetics*.

[24] Zhang Y., Huang C., Nie Y. (2021). Soluble CD163 is a predictor of mortality in patients with decompensated cirrhosis. *Frontiers in Medicine*.

[25] Groger M., Holnthoner W., Maurer D. (2000). Dermal microvascular endothelial cells express the 180-kDa macrophage mannose receptor in situ and in vitro. *Journal of Immunology*.

[26] Rodgaard-Hansen S., Rafique A., Christensen P. A. (2014). A soluble form of the macrophage-related mannose receptor (MR/CD206) is present in human serum and elevated in critical illness. *Clinical Chemistry and Laboratory Medicine*.

[27] Zou R., Gui X., Zhang J. (2020). Association of serum macrophage-mannose receptor CD206 with mortality in idiopathic pulmonary fibrosis. *International Immunopharmacology*.

[28] Gronbaek H., Rodgaard-Hansen S., Aagaard N. K. (2016). Macrophage activation markers predict mortality in patients with liver cirrhosis without or with acute-on-chronic liver failure (ACLF). *Journal of Hepatology*.

[29] Dai K., Huang L., Sun X., Yang L., Gong Z. (2015). Hepatic CD206-positive macrophages express amphiregulin to promote the immunosuppressive activity of regulatory T cells in HBV infection. *Journal of Leukocyte Biology*.

